The article "DNA hypermethylation of GDF5 in developmental dysplasia of the hip (DDH)" was published in 2019. Journal: Mol Genet Genomic Med.

# DNA hypermethylation of *GDF5* in developmental dysplasia of the hip (DDH)

**DOI:** 10.1002/mgg3.887

**Published:** 2019-07-23

**Authors:** Taghi Baghdadi, Mohammad Nejadhosseinian, Reza Shirkoohi, Reza Mostafavi Tabatabaee, Seyed S. Tamehri, Mojtaba Saffari, S. M. Javad Mortazavi

**Affiliations:** ^1^ Department of Orthopedic Surgery Tehran University of Medical Sciences Tehran IR Iran; ^2^ Joint Reconstruction Research Center Imam Khomeini Hospital, Tehran University of Medical Sciences Tehran IR Iran; ^3^ Department of Medical Genetics Tehran University of Medical Sciences Tehran IR Iran; ^4^ School of medicine Tehran University of Medical Sciences Tehran IR Iran; ^5^ Department of medical genetics, School of medicine Tehran University of Medical Sciences Tehran IR Iran

**Keywords:** Developmental Dysplasia of the Hip (DDH), DNA methylation, *GDF5*

## Abstract

**Introduction & Objective:**

Developmental Dysplasia of the Hip (DDH) is one of the most common congenital skeletal anomalies. Body of evidence suggests that genetic variations in *GDF5* are associated with susceptibility to DDH. DDH is a multifactorial disease and its etiology has not been entirely determined. Epigenetic changes such as DNA methylation could be linked to DDH. In this scheme, we hypothesized that changes in *GDF5* DNA methylation could predispose a susceptible individual to DDH.

**Methods:**

This study consisted of 45 DDH patients and 45 controls with healthy femoral neck cartilage, who underwent hemi‐, or total arthroplasty for the femoral neck fracture. A cartilage sample of 1 cm in diameter and 1 mm in the thickness was obtained for DNA extraction. DNA was extracted and DNA methylation of *GDF5* was evaluated by metabisulfite method.

**Results:**

Methylation analysis showed that the promoter of *GDF5* in cartilage samples from DDH patients was hypermethylated in comparison to healthy controls (*p* = .001).

**Conclusion:**

Our study showed that the methylation status of the *GDF5* in patients with DDH is dysregulated. This dysregulation indicates that adjustment in the methylation might modify the expression of this gene. Since this gene plays an essential role in cartilage and bone development, thus reducing its expression can contribute to the pathogenesis of DDH. Further studies are needed to elucidate the role of *GDF5* in this disease.

## 1 INTRODUCTION

Normal hip development relies on the femoral head and acetabulum development; the femoral head must be fixed in the hip socket to form concentrically and spherically. If the femoral head is not stable in its acetabulum, the hip joint undergoes developing incongruence and lack of sphericity. Most experts refer to looseness as subluxation or instability and dysplasia as physical deformity of the acetabulum and/or femoral head, but some authorities consider hip instability itself as dysplasia (Shaw & Segal, 2016). Hip dysplasia defines an abnormality in shape, size, organization or orientation of acetabulum, femoral head, or both. Shallow or immature acetabulum which is characterized as an acetabular dysplasia may lead to dislocation or subluxation of the femoral head. A dislocated hip is defined when there is no contact between the acetabulum and femoral head. The subluxed hip is a condition in which the femoral head is dislocated from its normal position but has its connection with acetabulum (Storer & Skaggs, 2006). DDH refers to a broad range of disorders with hip developmental problems from a hip with concentrically located, mild and stable dysplastic, to one with total dislocation and severe dysplastic (Aronsson, Goldberg, Kling, & Roy, 1994). Severe dysplasia is more likely to manifest clinically in early childhood or later infancy, whereas mild dysplasia might not become clinically apparent until adult life or might never present clinically at all (David et al., 1983).

The article "DNA hypermethylation of GDF5 in developmental dysplasia of the hip (DDH)" was published in 2019. Journal: Mol Genet Genomic Med.

The DDH incidence relies on various agents and is variable. The incidence for the dislocated hip is almost one in 1,000 live births and for hip subluxation is approximately 10 in 1,000 (Dezateux, Brown, Arthur, Karnon, & Parnaby, 2003; Lehmann, Hinton, Morello, & Santoli, 2000; Patel & Care, 2001). The incidence of all different types of DDH is probably higher but is not truly well known. The study by Rosendahl et al (Rosendahl et al., 2010) reported 1.3% prevalence of dysplastic but stable hips in general population. A study in the United Kingdom reported 2% prevalence of DDH in girls born in breech position (Bache, Clegg, & Herron, 2002). DDH is more common in girls than boys (Chan, McCaul, Cundy, Haan, & Byron‐Scott, 1997).

DDH risk factors generally are: postnatal environment, abnormal position in the third trimester, mechanical constriction of the fetus, and genetic predisposition. Risk factors related to intrauterine mechanical constraint are oligohydramnios, breech presentation, and large birth weight. These risk factors are very important in DDH development, but the mode of delivery of breech babies and breech presentation are the most important perinatal risk factor (Chan et al., 1997; Lapunzina, Camelo, Rittler, & Castilla, 2002; Wald, Terzian, Vickers, & Weatherall, 1983). Tight swaddling and use of cradle boards, postnatal swaddling practices lead to long periods of adduction and extension of thighs significantly associated with high rates of DDH (Salter, 1968; Yamamuro & Ishida, 1984). Modern caring methods such as the use of very slim disposable nappies and baby seats for a long time could be associated with DDH. Maternal hormonal milieu may lead to joint laxity which predisposes babies to DDH, but there is no association with change in concentration levels of serum beta‐estradiol, urinary estrogen, and serum or cord blood relaxin (Forst, Forst, Forst, & Heller, 1997; Thieme, Wynne‐Davies, Blair, Bell, & Loraine, 1968).

The article "DNA hypermethylation of GDF5 in developmental dysplasia of the hip (DDH)" was published in 2019. Journal: Mol Genet Genomic Med.

Genetic involvement in DDH risk is more evident than past. Between 12 and 33 percent of DDH patients have a positive family history (BJERKREIM, ÅRSETH, & Palmén, 1978; Haasbeek, Wright, & Hedden, 1995). It has been reported that when one sibling is affected, the risk for DDH development is 6 percent, the risk with one affected parent is 12 percent, and the risk would be 36 percent if one sibling and one parent are affected (Wynne‐Davies, 1970). If one monozygotic twin is affected, the risk for another twin would be about 40 percent (S Jay Kumar, 1988). Recent studies have shown that the risk of DDH for familial relatives is high, with first‐degree relatives having 12 times more at risk of DDH development than controls (Carroll et al., 2016; Schiffern et al., 2012; Stevenson et al., 2009).

The genetic implication in DDH development is not all the story, 40% concordance rate for DDH in identical twins highlights the important role of epigenetic and environmental factors in DDH pathogenesis. DDH is a multifactorial disorder in which both genetics and nongenetic factors are implicated. Nevertheless, the exact mechanisms of DDH pathogenesis are not understood. Epigenetics is a process which influences gene expression without any changes in DNA sequences. DNA methylation is one of the epigenetic mechanisms which is controlled by DNA methyltransferase (DNMT) enzymes. DNMT enzymes transfer the methyl group (CH_3_) onto the cytosine residues to form a 5‐methylcytosine (Jones, 2012). DNA methylation through two mechanisms leads to chromatin remodeling and gene suppression, first is mediated directly by the inhibition of transcription factors binding to DNA and second is mediated through proteins with methylated DNA binding domain (MBD) which creates links between histone proteins and methylated DNA (Greer & McCombe, 2012).

Growth Differentiation Factor 5 (*GDF5*) is a member of transforming growth factor beta (TGF‐β) superfamily and is implicated in the repair and maintenance of synovial joints (Luyten, 1997). This gene is also paly roles in chondrocyte proliferation and chondrogenesis (Buxton, Edwards, Archer, & Francis‐West, 2001; Francis‐West et al., 1999; Nakamura et al., 1999). *GDF5* (OMIM: 601146) plays an important role in normal development of bone and joint (Settle Jr et al., 2003). *GDF5* mutations are linked with various rare skeletal disorders such as type A2 and type C of brachydactyly (Polinkovsky et al., 1997; Seemann et al., 2005), grebe type of chondrodysplasia (Thomas et al., 1997), Hunter‐Thompson type of acromesomelic dysplasia, (Thomas et al., 1996), and DuPan syndrome (Faiyaz‐Ul‐Haque et al., 2002).

The article "DNA hypermethylation of GDF5 in developmental dysplasia of the hip (DDH)" was published in 2019. Journal: Mol Genet Genomic Med.

Many studies reported that *GDF5* is involved in DDH pathogenicity (Dai et al., 2008; Rouault et al., 2010; Zhao et al., 2013). We aimed to evaluate the role of DNA methylation of the *GDF5* in DDH pathogenesis. In this study, the methylation profile of *GDF5* has been assessed. Based on our knowledge, this is the first study which provides information about *GDF5* methylation pattern in DDH and results of this study could be useful in diagnosis and might provide promising therapeutic tool in the future.

## 2 MATERIAL AND METHODS

### 2.1 Patients and controls

Patients were enrolled after DDH diagnosis at the orthopedics clinic of Imam Khomeini Hospital of Tehran University of medical sciences. A control group who did not have DDH, metabolic bone disease, or osteoarthritis was also recruited in the study at the same time. The study consists of a total of 90 ancestry individuals (45 DDH patients and 45 healthy controls with Mean age ± *SD* of 45 ± 12.6 and 42 ± 15.2 respectively). The patient group consisted of five males and 40 females. The healthy controls also consisted of five males and 40 females, and they had neither family history nor clinical evidence of any inflammatory disorders and arthritis. The control sample taken from individuals with healthy femoral head cartilage which due to fracture of the femoral head were underwent a hemi‐, or total hip arthroplasty operation. Informed consent was taken from all controls and patients. The Human Research Ethics Committee of Tehran University of Medical Sciences approved this study.

### 2.2 Tissue collection

Cartilage samples were taken from the femoral head of DDH patients and healthy individuals. Genomic DNA was extracted from cartilage tissues using the QIAamp DNA Mini Kit (Qiagen) according to manufacturer's instruction. Extracted DNA samples were stored at −20 C. Quantification of DNA samples was determined at 260 and 280 nm by spectrophotometry (NanoDrop 2000c Spectrophotometer, Thermo Fisher Scientific, Wilmington, DE, USA).

### 2.3 DNA treatment through bisulfite conversion

Genomic DNA from cartilage tissue samples were extracted and treated with bisulfite (EpiTect Plus DNA Bisulfite Kit) which converts unmethylated cytosine to uracil, whereas methylated cytosines are unaffected. Before starting, the following notes were considered.

The article "DNA hypermethylation of GDF5 in developmental dysplasia of the hip (DDH)" was published in 2019. Journal: Mol Genet Genomic Med.

Thirty milliliters ethanol (96%–100%) was added to Buffer BW and stored at room temperature (15–25°C), 27 ml ethanol (96%–100%) is added to Buffer BD and stored at 2–8°C, 310 μl RNase‐free water is added to carrier RNA and stored in aliquots at –20°C.

### 2.4 EpiTect Plus DNA Bisulfite Kit, Quick‐Start Protocol

#### 2.4.1 Protocol 1, Bisulfite conversion of DNA

Eight hundred microliters RNase‐free water was added to each aliquot of Bisulfite Mix and vortexed until Bisulfite Mix was completely dissolved which might take up to 5 min. Bisulfite reactions in 200 μl PCR tubes were applied according to protocol. PCR tubes were closed and bisulfite reactions were mixed thoroughly. After mixing the reactions, blue color of the DNA Protect Buffer indicating sufficient mixing and correct pH. Thermal cycler program was set up according to the protocol. PCR tubes were placed in the thermal cycler and incubated.

#### 2.4.2 Protocol 2, Cleanup of converted DNA

For starting material <100 ng DNA, dissolved carrier RNA was added to Buffer BL. Upon completion of bisulfite conversion in protocol 1, PCR tubes were briefly centrifuged and reactions were transferred to 1.5 ml microcentrifuge clean tubes. According to protocol 2, 310 μl Buffer BL (with 10 μg/ml carrier RNA for <100 ng DNA) was added to each sample. Mixed by vortexing and then centrifuged briefly. Two hundred and fifty microliters ethanol (96%–100%) was added into each sample. Mixed by pulse vortexing for 15 s and then centrifuged briefly to remove drops from inside the lid. MinElute DNA spin columns and collection tubes were placed in a rack. The entire contents of each tube was transferred to a corresponding spin column. The spin columns were centrifuged at maximum speed for 1 min. The flow‐through was discarded and placed the spin columns back into the collection tubes. 500 μl Buffer BW was added to each spin column and centrifuged at maximum speed for 1 min. The flow‐through was discarded and the spin columns were placed back into the collection tubes. Five hundred microliters Buffer BD was added to each spin column, the spin column lids were closed, and incubated for 15 min at room temperature (15–25°C). The spin columns were centrifuged at maximum speed for 1 min. The flow‐through was discarded and the spin columns were placed back into the collection tubes. Five hundred microliters Buffer BW was added to each spin column and was centrifuged at maximum speed for 1 min. The flow‐through was discarded and the spin columns were placed back into the collection tubes. The previous step was repeated. Two hundred and fifty microliters ethanol (96%–100%) was added to each spin column and centrifuged at maximum speed for 1 min. The spin columns were added into new 2 ml collection tubes and centrifuged at maximum speed for 1 min to remove any residual liquid. The spin columns were incubated on a heating block at 60°C for 5 min to evaporate the liquid. The spin columns were placed in 1.5 ml microcentrifuge clean tubes. Fifteen microliters Buffer EB was directly added to the center of each spin column membrane and lids were closed gently. The spin columns were incubated at room temperature for 1 min and centrifuged for 1 min at 15,000*g* (12,000 rpm) to elute the DNA. The purified DNA was stored at 2–8°C for up to 24 hr. For longer storage, it was recommended to store at –20°C.

The article "DNA hypermethylation of GDF5 in developmental dysplasia of the hip (DDH)" was published in 2019. Journal: Mol Genet Genomic Med.

### 2.5 PCR amplification

The DNA target for PCR amplification was constituted of a 178 base pair segment at 20q11 band that was part of a CpG island from the promoter region of *GDF5* (NM_000557.5). The mentioned segment was selected in targeted DNA using UCSC (University of California, Santa Cruz) website (https://genome.ucsc.edu/). Primers were designed by Methprimer database (http://www.urogene.org/cgi-bin/methprimer/methprimer.cgi). For PCR amplification, each tube contained variable (maximum 20 μl) of bisulfite‐treated DNA, 85 μl of bisulfite mix, 35 μl of DNA Protect Buffer, variable RNase‐free water with total volume 140 μl. The combined volume of DNA solution and RNase‐free water was 20 μl for high concentration samples (1ng – 2 μg). The amplification conditions for PCR cycles were as follows: denaturation at 95°C for 5 min, incubation at 60°C for 25 min, denaturation at 95°C for 5 min, incubation at 60°C for 85 min (1 hr 25 min), denaturation at 95°C for 5 min, incubation at 60°C for 175 min (2 hr 55 min). After PCR amplification, all samples were gel electrophoresed for amplification validation and afterward sequenced (Macrogen) and the results were analyzed by Codon Code Aligner version 2 (Codon Code Corporation) software.

### 2.6 Statistical analysis

Data analysis was performed using SPSS software version 23 (SPSS, Chicago, IL, USA). The Kolmogorov–Smirnov test was applied to evaluate the normality of the variables. Based on our data, whether normally distributed or not, independent sample *t*‐test and Mann–Whitney test were applied, respectively. In order to draw graphs, GraphPad Prism version 5 for windows (GraphPad Software, www.graphpad.com) was applied. All results are expressed as mean ± S.D. with statistical significance set at 0.05.

## 3 RESULTS

### 3.1 Methylation level of *GDF5* promoter

Methylation status of *GDF5* promoter in DDH patients and healthy controls is shown in Figure 1 and Table 1. In overall view, methylation analysis showed that the promoter of *GDF5* in cartilage samples from DDH patients was hypermethylated in comparison to healthy controls (*p* = .001, Figure 1, Table 1).

The article "DNA hypermethylation of GDF5 in developmental dysplasia of the hip (DDH)" was published in 2019. Journal: Mol Genet Genomic Med.

**Figure 1:** Methylation status of GDF5 promoter in DDH patients and healthy controls

**Table 1:** Methylation status of *GDF5* promoter in DDH patients and healthy controls

***GDF5***	**Groups**		***p*‐value**
	DDH	Healthy	
Methylated	33 (73.3)	1 (2.2)	**.001**
Unmethylated	12 (26.7)	44 (97.8)	
Total	45 (100)	45 (100)	

## 4 DISCUSSION

Developmental dysplasia of the hip is a complex disorder that genetic and nongenetic factors are involved in its etiology. It is known that environmental factors such as breech position, female sex, tight swaddling and use of cradle boards, and oligohydramnios are associated with the development of DDH (Shaw & Segal, 2016). The high concordance rate in monozygotic twins compared to dizygotic twins and a 12‐fold increase in DDH among first‐degree relatives indicates that genetic has an important role in the disease, however, it also indicates that genetics solely cannot cause the disease (Stevenson et al., 2009; Weinstein, 1987). It seems DDH is a multifactorial disease with genetic and epigenetic causes, only genetics cannot solely lead to the disease, and epigenetic factors might contribute to the disease.

Currently, interests have been drawn toward the collaboration and interaction between genetic and environmental factors that finally impress the epigenome (Mahmoudi, Aslani, Nicknam, Karami, & Jamshidi, 2017; Quaden, De Winter, & Somers, 2016). Considering these facts, to explain the etiology of DDH, epigenetics has a unique importance. Although we could not find any methylation studies about the evaluation of *GDF5* in the field of DDH disease, but previous studies showed that *GDF5* promoter in osteoarthritis (OA) patients is regulated by methylation (Reynard, Bui, Canty‐Laird, Young, & Loughlin, 2011; Reynard, Bui, Syddall, & Loughlin, 2014). These abovementioned studies suggested that the dysregulation of *GDF5* expression through altered methylation level would probably contribute to OA development. Nonetheless, there were no other studies to evaluate DNA methylation of *GDF5* in DDH. This study showed that different methylation pattern can be detected in healthy control and DDH patients.

*GDF5* is a member of TGF‐β (transforming growth factor beta) superfamily and is implicated in the repair and maintenance of synovial joints (Luyten, 1997), chondrocyte proliferation, and chondrogenesis (Buxton et al., 2001; Francis‐West et al., 1999; Nakamura et al., 1999). It has been evident that *GDF5* is important for normal skeletal, joint, and bone development (Settle Jr et al., 2003), as well as *GDF5* mutations lead to various rare skeletal diseases (Faiyaz‐Ul‐Haque et al., 2002; Polinkovsky et al., 1997; Seemann et al., 2005; Thomas et al., 1997, 1996).

The article "DNA hypermethylation of GDF5 in developmental dysplasia of the hip (DDH)" was published in 2019. Journal: Mol Genet Genomic Med.

*GDF5*, which is located on human chromosome 20q11.22, encodes a secreted ligand of the TGF‐β superfamily of proteins. Binding of TGF‐β ligands to different TGF‐β receptors results in recruitment and activation of transcription factors family called SMAD which changes the expression of downstream genes. *GDF5* regulates the development of various cell types and tissues, such as joints, teeth, cartilage, brown fat, and the growth of dendrites and neuronal axons. Mutations in *GDF5* are associated with various skeletal disorders such as brachydactyly, proximal symphalangism, acromesomelic dysplasia, multiple synostoses syndrome, chondrodysplasia, and susceptibility to osteoarthritis (Enochson, Stenberg, Brittberg, & Lindahl, 2014; Francis‐West et al., 1999; Polinkovsky et al., 1997; Ratnayake et al., 2017; Thomas et al., 1997, 1996).

Furthermore, *GDF5* is involved in the development of the embryonic organs, especially it has an important role in the formation of the articular cavity and articular cartilage. *GDF5* also implicates in the early stages of skeletal development, adhesion and clustering of chondrocyte cells. In the later stages, *GDF5* also involves in hypertrophy and proliferation of the cartilage cells. This gene is expressed in the cartilage and plays roles in bones and joints development. Studies documented that mutations in *GDF5* lead to an increased risk of arthritis, short bones, and skeletal disorders (Dai et al., 2008; Lettre, 2017; Plett, Berdon, Cowles, Oklu, & Campbell, 2008; Rouault et al., 2010; Zhao et al., 2013). According to these body of evidences, *GDF5* is an appropriate candidate gene for the evaluation of articular and bone abnormalities.

Evaluation of *GDF5* methylation in DDH has not been performed so far, and only two studies have evaluated the methylation of this gene in OA patients, both of which have shown that the expression of this gene is regulated by methylation (Reynard et al., 2011, 2014).

In this study, we showed that the *GDF5* was significantly different in terms of methylation between the patient and control groups and the methylation status of *GDF5* in the patient group was significantly higher than healthy controls and this increase in methylation could lead to decreased expression of the gene. Since this gene plays an important role in the development of joints and bones, high methylation status which resulted in a reduced expression might lead to defects in bone and cartilage formation and eventually skeletal diseases such as DDH. More studies are needed to determine the role of this gene in the DDH development, and it is possible that the DNA methylation of *GDF5* might use as a diagnostic and prognostic marker.

The article "DNA hypermethylation of GDF5 in developmental dysplasia of the hip (DDH)" was published in 2019. Journal: Mol Genet Genomic Med.

Our study had several important limitations. First of all, it is not completely clear whether all of these epigenetic modifications such as DNA methylation are actually caused by disease or a consequence of the disease. All DDH patients were at late stage of the disease. Since there is a chronic inflammation in the joints, one theory is that the chronic inflammation and proinflammatory cytokines are the main cause of these abnormalities in DNA methylation. Therefore, further study to compare the methylation signature in early and late stages of DDH patients is essential, though, this is not an easy study to be done. Second, we could not explain why this epigenetic silencing of the *GDF5* only affects the hip joint and not the other joints. One possible explanation is that the DDH is a multifactorial disease and its epigenetic silencing would be a factor that could play a role.

In conclusion, epigenetic alterations could be considered as a helpful diagnostic and follow‐up marker in DDH and might be a promising therapeutic tool in the future. Hopefully, improving our knowledge about the epigenetic modifications that happen in the DDH development increases the prospects for controlling or preventing DDH abnormalities. In this regard, we identified that there is a difference in the methylation status of *GDF5* promoter in the cartilage tissue of DDH patients in comparison with healthy controls. Although specific effects of *GDF5* methylation during this disease require further investigation, we suggest that hypermethylation of *GDF5* may contribute to the DDH pathogenesis.

## CONFLICT OF INTEREST

The authors declare no conflict of interest.
